# Nutraceuticals: Pharmacologically Active Potent Dietary Supplements

**DOI:** 10.1155/2022/2051017

**Published:** 2022-07-04

**Authors:** Subhash Chandra, Sarla Saklani, Pramod Kumar, Bonglee Kim, Henrique D. M. Coutinho

**Affiliations:** ^1^Department of Pharmaceutical Chemistry, School of Sciences, Hemvati Nandan Bahuguna Garhwal (A Central) University, 246174, Srinagar Garhwal, Uttarakhand, India; ^2^Department of Pharmaceutical Sciences, HNB Garhwal University, Srinagar Garhwal, India; ^3^College of Korean Medicine, Kyung Hee University, Seoul 02447, Republic of Korea; ^4^Department of Biological Chemistry, Regional University of Cariri (URCA), Crato, Brazil

## Abstract

A growing demand exists for nutraceuticals, which seem to reside in the grey area between pharmaceuticals and food. Nutraceuticals, up today, do not have a specific definition distinct from those of other food-derived categories, e.g., food supplements, herbal products, functional foods, and fortified foods. They have, however, a pharmacological beneficial effect on health. Many studies have been recently addressed to assess their safety, efficacy, and regulation. The object of writing this review article is that we need to pay more attention to natural and organic foods. The bases of nutraceutical components (food supplements) are known for potent and powerful clinical evidence effects on the treatment of hypertension and type 2 diabetes.

## 1. Introduction

Nutraceutical use is growing fast and is well accepted by people for its all-natural origin. Nutraceuticals cannot replace pharmaceuticals but can be used in the prevention and cure of some pathological conditions. According to Stephen DeFelice (1989), a nutraceutical is a food or part of food capable of providing beneficial health effects, including the prevention and the treatment of disease, which is not applicable to food supplements [1]. Nutraceuticals are obtained from foods of plant or animal origin, and worldwide research focused on their mechanism of action, safety, and clinical data. These are therapeutic agents that do not propose themselves as an alternative to drugs but instead can be helpful to prevent a cluster of conditions that could occur together (metabolic syndrome), e.g., type 2 diabetes, stroke, heart disease, and cardiovascular disease. Nutraceuticals are a challenge for the future of prevention and therapy and a triggering tool in the medicine area. The possibility of preventing or supporting a pharmacological treatment, which is nowadays mainly based on pharmaceuticals, can be a powerful tool to face pathological, chronic, and long-term diseases in subjects who do not qualify for pharmacological therapy [2].

The excessive demand for natural healthcare has dramatically improved the price of hospital treatment, so humans have used herbal nutritional food, dietary supplements, and nutraceuticals for the usage of phytotherapy or nutritional therapy to replace or get rid of radiotherapy or chemotherapy [3]. This superior and practical know-how had been assisted to standardize production methods and clinical practices for nutraceutical markets. The Indians, Chinese, Japanese, Egyptians, and Sumerians have provided clinical evidence, suggesting that nutraceutical or food supplements can be efficaciously used as remedies to treat/prevent exclusive forms of ailment [4]. Nutraceutical food affords better fitness with greater benefits, which claims to prevent subacute and continual ailment and improve fitness with put off the getting older technique and boom lifestyle expectancy [5].

The term nutraceutical is largely used to indicates the usage and effectiveness of a variety of herbal products [6]. The “nutritional elements” products are herbs, vitamins, proteins, minerals, fat, fiber, and amino acids) (Tables 1 and 2). The dietary meal nutrient ingredients can be collections, isolates, or concentrates and may be found in lots of stages along with tablets, capsules, suspension and emulsion drugs, soft gel, gel cap, suspension, emulsion, drinks, or powders [7]. The nutritional meal complement, including the vitamin B complement, is normally sold in pill shape. The nutraceuticals are broadly utilized in human fitness, e.g., cancer treatment, Vita. E, Vita. D, soy, green tea, selenium, and lycopene (Table 2), which describe nutraceuticals as meals or nourishment supplements that produce medical or fitness advantages, inclusive of the prevention/treatment of any type of sickness [8].

This special issue is dedicated to the role and perspectives of nutraceuticals in human health, examined from different angles, ranging from analytical aspects to clinical trials and from efficacy studies to beneficial effects on health conditions.

### 1.1. Sources and Methodology

The literature data was collected via Core Collection, Web of Science, Google Scholar, Scopus, Science Direct, PubMed, MDPI, Clarivate Analytical, Google Academic, and Scientific Electronic Library Online (SciELO) from 1990-21. The search terms were nutraceuticals, food supplements, medicinal food, and functional food. These articles were considered on the basis of their nutraceutical and therapeutical uses with scientific proof.

## 2. Nutraceutical Hypothesis

These are based on the meal assets, MOA, useful food, chemical nature [9, 10], fatty acids, dietary fiber, proteins, vitamins, minerals, carbohydrates, spices, probiotics, prebiotics, polyunsaturated fatty acids, polyphenols, amino acids, antioxidants, antimicrobial, antidiabetic, analgesics, anti-inflammatory, carotenoids, dairy-primarily based elements, nutritional lipids, oils, phytochemicals, plant extracts, peptides, soy-primarily based substances, and premixes.

Essentially, the nutraceuticals are mainly categorized into two elements [11].

1. Potential nutraceuticals
2. Established nutraceuticals [12]

### 2.1. Functional Ingredients

Functional foods are typically classified as traditional foods that have been enriched with an ingredient (bioactive in many cases) that is able to provide additional benefits to human health. Functional foods are those ingredients that are used after clinical intelligence and knowledge. They have used especially healthy life and more resistant survival [13]. Functional foods are fed on to eat evidently as opposed to any dosage form as alike tablet, tablet, and liquid dosage form. On occasion, extra complementary nutrients are covered, which include vitamin D in milk. The Canadian health organization describes or outlines approximately functional foods, the ones are “regular meals that have components or elements introduced to offer it a selected scientific or physiological advantage, apart from a merely dietary effect.” According to Japan, all practical ingredients must be present and occurring of their herbal shape [14] in place of a tablet, capsule, and powder [15] consumed in the food plan as every so often or every day [16] and ought to modify a biological system in wish of preventing/controlling disease or disorder-like situations [17].

### 2.2. Medicinal Foods

The medicinal or clinical foods are not present as a chip consequence to clients. The “Food & Drug Administration” contemplates medical nourishment to be “formulated, to be fed on or administered internally under the supervision of a physician and which is meant for the particular nutritional control of a disease or circumstance for which one-of-a-kind dietary necessities, on the idea of recognized scientific ideas, are established by way of medical evaluation.” The clinical food ingredients are designed to satisfy nutritional requirements for humans identified or observed out with unique contamination and ingested through oral or tube feeding. These ingredients are regulated by using FDA and authorized by scientific direction.

## 3. Phytochemicals as Nutraceutical Ingredients

Plants comprise primary and secondary metabolites, which showed and play various styles of functions. The primary metabolites, which play a vital position in mobile strategies, may be simple sugar, carbohydrates, nucleic acids, lipids, and amino acids. Secondary metabolites are used in pressure and deterrent. Plants grow and expand the special varieties of secondary metabolites, which can be used in beneficial positions for people and residing organisms. Its miles are referred to as plant herbal products (Figures 1 and 2).

### 3.1. Carotenoids

The carotenoids are observed in exceptional colorings and nature, e.g., carrots orange, corn yellow, tomato red, salmon, flamingos, goldfish, and autumn leaves, while “chlorophyll” has gone via the leaves, simplest carotenoids and phenols continue to be. The bell peppers of various colorations offer a ramification of various carotenoids:

*Orange carotenoids*: alpha, beta, and gamma carotene.

*Red carotenoids*: lycopene and astaxanthin.

*Yellow carotenoids*: lutein and zeaxanthin.

Plants produce more than six hundred carotenoids, and the handiest 50 carotenoids in the human weight-reduction plan are absorbed into the bloodstream. The *α*, *β*, and some other carotenoids (“not lycopene or lutein”) may be transformed to vitamin A. Hypervitaminosis of vitamin A cannot be because of immoderate *α*- and *β*-carotene intakes since the switch and absorption rates are too gradual. Each of the carotenes (*α*-carotene and *β*-carotene) is protecting against liver and lung cancers in the cell way of life and animal research. The most lipid-rich (LDL) cholesterol particles are transported by means of carotenoids into blood movement and get hold of the maximum LDL receptors.

### 3.2. Lycopene

Lycopene is found in watermelon, tomatoes, pink grapefruit, papaya, and guava and additionally offers red color. It is a potent antioxidant compound that reduces damage to DNA and proteins and additionally offers better pores and skin safety in opposition to extremely violet light than *β*-carotene. It is utilized in most cancer protection and decreases LDL levels of cholesterol and suppresses insulin-like increase elements, which stimulates tumor boom.

### 3.3. *β*-Carotene

*β*-Carotene is a much less lively antioxidant, however robust in opposition to singlet oxygen, their components can fairly enrich *β*-carotene content and LDL cholesterol without affecting different carotenes, they are able to increase the pastime of herbal killer “T-cells, *β*-cells, and NK cells,” and energizing “DNA” mend enzymes and grant higher cornea safety in opposition to extremely violet light than lycopene.

### 3.4. *α*-Carotene

*α*-Carotene is 10 instances stronger and a more effective anticarcinogenic compound in assessment than *β*-carotene, because of the let out of immunogenic cytokines (IL-1 and TNF-*α*).

### 3.5. Lutein

Lutein produces yellow color in nature through the exceptional types of resources, e.g., corn, avocado, and egg yolk. It protects and therapies the attention, from macular degeneration and cataracts, which shield against colon cancer. Its maximum concentration or quantity is located in kale, spinach, watercress, and parsley.

### 3.6. Astaxanthin

Astaxanthin gives different colors to salmon, shrimp, and crab. It is a potent antioxidant rather than any other carotenoid. It is also improved T-cell manufacturing and cytokine, which releases and crosses the “blood-brain barrier” (BBB) brain antioxidant and authorizes it to liberate trapped absolutely to vitamin C.

### 3.7. Saponins

Saponins are a legume's own family medicinal plant, the ones that occur in chickpeas and soybeans and eliminate LDL cholesterol. They are effective in opposition to colon cancers and a few other crucial troubles.

### 3.8. Terpineol

Terpineol produces carrot flavor from carrots, and the origin cellular pattern is detained in most cancer stalls. They are water-insoluble chemical compounds, classified as hydrocarbon constituents by isoprene units and a high class of secondary metabolites [18, 19]. It is used in exhibiting antimicrobial and cytotoxic potential [20, 21].

### 3.9. Limuloids

Limuloids are present in orange membranes and peels, which are 45 times more potent anticarcinogenic than hesperidins. It detoxifies cancer agents and promotes most cancers' cellular apoptosis, one-limonene smells “piney” like turpentine, d-limonene smells like orange, and it is able to be used as a solvent and cleanser.

### 3.10. Anthocyanins

Anthocyanins are water-soluble, anti-inflammatory glycosides and acryl-glycosides; they make roses red, cherries, strawberries, blueberries, and violet-blue. Blueberries increase anthocyanin contents when ripened and are easily damaged by heat (cooking).

### 3.11. Flavonoids

Flavonoids (flavone-like) are antioxidant and anti-inflammatory nature chemical compounds, which are present in dark chocolate and red wine and absent in white wine, due to their different extraction methods, where red wine is prepared or made by the fermentation method, although ultrafiltration is every now and then used to reduce astringency and bitterness. It is used for those patients, who are suffering from radiation and chemotherapy [22].

### 3.12. Ruthin

It is determined in asparagus, buckwheat, and citrus quit end result, which is not misplaced in drying grapes to raisins and strengthens arteriole partitions.

### 3.13. Quercetin

Quercetin (“flavanol”) which is the mighty antioxidant is present in green tea, red onions, buckwheat, and red grapes, which is distinctly available in the skins of apples and decreases LDL oxidation and is a vasodilator and blood thinner and might kill viruses. It is used to relieve allergy, inhibit catechol-O-methyl transferase (COMT) enzymes, reduce epinephrine, inhibit heart stroke protein and antihistaminic activity, and also promote apoptosis in cancer and other cells.

### 3.14. Tannins

Tannins (polyphenolics) are used to tan and defend leather-based seen in the 18th century A.D., which makes cranberries and pomegranates sour. It together with vitamin C helps to construct and improve collagen. It prevents UTI (“urinary tract infection”) with the useful resource of stopping microorganisms (bacteria) from adhering to the partitions. While blended with anthocyanins (“as in pomegranate juice”), it damage down oxidized LDL cholesterol within the bloodstream and in the atherosclerotic plate. It available in maximum energetic shape is black tea, which includes 90% catechin and epicatechin in natural grapes.

### 3.15. Phenolic Acids

The phenolic compounds (proanthocyanidins, resveratrol, and ellagic acid) are found in red wine, grape juice, and raisins, which are fantastically found in cranberry juice, reducing oxidation of LDL cholesterol and adherence of bacteria to enamel/teeth and cellular lining of the bladder, thereby lowering UTI (“urinary tract infections”) and tooth fairy. The sugar-coat nature compounds lessen the nonstick homes of phenolic. The phenolic acid formation of most cancers sells nitrosamines from dietary nitrate and nitrites.

### 3.16. Ellagic Acid

Ellagic acid is determined in strawberries and raspberries but is 50% greater in raspberries; it reduces esophageal and colorectal cancers, which retard the process of DNA adducts, retard stage 1, and potentiate phase-2 adjuvant.

### 3.17. Chlorogenic Acid

Chlorogenic acid is present in high excessive amounts in blueberries, tomatoes, and bell peppers, alongside the ester of caffeic acid (“hydroxyl cinnamic acid”), which diminish mutagenicity of polycyclic fragrant hydrocarbons and showed potent antioxidant activity.

### 3.18. Ferulic Acid

Ferulic acid is plentiful inside the cellular walls of seeds of whole wheat, brown rice, oats, apple, artichoke, orange pineapple, and peanut. Its miles are used as an antioxidant and anticancer, a precursor to vanillin and antitumor activity in breast and liver cancers.

## 4. Dietary Supplements

On the premise of the US (“DSHEA”) “Dietary Supplements Health & Education Act” 1994, the nutritional additives are those that include fatty acids, fiber, protein, vitamin, amino acid, and mineral, which are referred to as dietary ingredients or dietary supplements [6, 23].

LCPUFAs are crucial for foetal and infant growth and development because of their essential position in cellular growth and biotransformation or metabolism, membrane shape, and function [24]. The LCPUFAs (“flaxseed, flaxseed oil, walnuts, canola oil, and soybean oil”) result in brain growth and irrevocable damage due to both of them being wealthy in arachidonic acid and docosahexaenoic acid, primarily based on the clinical evidence and epidemiology that dietary *ω*-3 type polyunsaturated fatty acid decreases the risk of heart ailment [25]. The main five essential fatty acids for human consumption are saturated palmitic acid, stearic acid, monounsaturated oleic acid, polyunsaturated linoleic, and linolenic acids [26]. The newly synthesized secure, less expensive, and sustainable plant origin of these fatty acids is arachidonic acid, eicosatetraenoic acid, and docosahexaenoic acid [27]. Today's and greater currently eicosatetraenoic acid and docosahexaenoic acid were fabricated in *Brassica juncea* with an excessive capitulate [28].

### 4.1. Amino Acids

The amino acids are playing a significant role in anti-inflammatory, immunomodulatory, and antioxidant properties [29]. These are used in protein biosynthesis and many others, e.g., L-arginine is used for infant or children growth, pregnant women, and synthesis of agmatine, urea, creatine, polyamines, and nitric oxide. It is also useful for antihypertensive and antiproliferative effects on vascular smooth muscles. Glutamine is essential for metabolic stress, burn injury, muscle wasting, weight loss, and other infections with depletion of plasma. It has been shown to gain patients and decreases the mortality rate [30] by elevating the level of amino acids in staple meals which include rice, wheat, corn, and different flora [16, 31].

## 5. Micronutrients

### 5.1. Vitamins

These are micronutrients/food supplements, which play a significant role in our daily life for better health and are essential for metabolic pathway, as an enzyme cofactor forerunner [32].

### 5.2. Minerals

Minerals are those chemical compounds which are vital for the normal growth and development of all residing organisms (humans, animals, and plants). They protect our bodies from various types of diseases. A right and healthy amount of mineral intake/consumption is crucial to maintaining an exact diet nutritionally, which will reduce the major disease such as cardiovascular and degenerative disease, diabetes, digestive disorder, and cancer [33, 34] (Table 3).

## 6. Nutraceuticals as Clinical Study

### 6.1. Healthy Fats (MUFA *ω*-9 and PUFAs *ω*-3 and *ω*-6)

Monounsaturated fatty acids and polyunsaturated fatty acids are linked or connected with a reduced chance of coronary heart disease [35].

### 6.2. Monounsaturated Fatty Acids (MUFA/*ω*-9)

On the basis of 7 nations' statistics, the death rate from “CHD” became specifically low in Mediterranean nations, wherein the olive oil has been used, which is exceedingly enhanced with MUFA and fats. The protective impact of MUFA in competition with CHD became additionally supported via using a retrogression investigation of information from the “nurse health” look at of 80082 females observed for much less than 14 years and additionally found a fantastic affiliation amongst consumption of MUFA and CHD danger [36–38]. We have got presently stated in asymptomatic excessive cardiovascular chance topics that consumption of traditional Mediterranean weight-reduction plan augmented with virgin olive oil actively regulates the articulation of lead chromosome concerned in vascular irritation, foam cell process, and thrombosis inside the course of an antiatherothrombotic profile [39].

### 6.3. Polyunsaturated Fatty Acids (PUFAs)

ALA (“*α*-linolenic acid”) and LA (“linoleic acid”) belong to the *ω*-three (“omega-3”) and *ω*-6 (“omega-6”) collection of PUFA separately. The resources of omega three and omega six are seafood and fatty fish, optimum vegetable oils, grains, and walnuts. PUFA omega-three fatty acids show potent primary and secondary prevention or cure of cardiovascular disorder [40]. Polyunsaturated fatty acids are traditionally useful for human health [41, 42] which is based on the two types of omega-3 and omega-6 series. The health benefit of the *ω*-three and *ω*-six ratio in macroalgae allows their use in the method of practical meals and convenience food. These fatty acids lessen the possibility of chest, colon, prostate, and renal cancers, and other effects are suppressing inflammation, asthma, and rheumatoid arthritis [43]. It is especially used in cardiovascular and inflammatory diseases and skin health [44].

### 6.4. Cholesterol Reduction

All agents reduce LDL cholesterol absorption in the intestinal gut and additionally reduce plasma LDL concentrations. A metaevaluation of forty-one trials showed that consumption of 2 gm/day of stanols or sterols decreased LDL concentration by using about ten-eleven% [45]. The “American Heart Association” and “European Current Dietary Guideline” aid plant sterols as a healing option for people with improved levels of cholesterol [46, 47]. In a pooled evaluation of ten prospective cohorts, each 10 gm/day increment of energy-adjusted general nutritional fiber becomes associated with a 14% lower hazard of coronary activities and a 27% decrease in the hazard of coronary loss of life [48].

### 6.5. Coenzyme Q-10 (CoQ-10)

CoQ-10 is an herbal food substance, and its miles are used for functional food and dietary supplements. It is an internal lipophilic substance, which is a crucial or useful substance of mitochondrial strength biotransformation and additionally effective for antioxidants and effective for human fitness [49–51]. CoQ-10 limited deterioration of viscoelasticity and reduce the wrinkle 7 microrelief lines and improved/increased skin smoothness/fairness.

## 7. Effectiveness and Safety

### 7.1. Regulatory Aspects

The regulation of nutraceuticals presents a noteworthy challenge to the globalization of nutraceuticals, with a murky and somewhat dissimilar definition of these products that are used in different countries. In general, the goals of nutraceutical regulation have been focused on safety and labeling with a lesser emphasis, as compared to pharmaceuticals, on product claims and intended use. The first step in food regulation in Europe was established in 1997 with the Green Paper after that the safety and use of food were set by the United Nations Food and Agricultural Organization (FAO) and the World Health Organization (WHO) in the *Codex Alimentarius* (FAO/WHO1992). In the USA, the FDA, which focuses on safety aspects and food supplements, acknowledges the term nutraceutical and applies a different set of regulations to them than those of conventional foods and drugs. As per the Dietary Supplement Health and Education Act established in 1994 (DSHEA), it is the manufacturer's responsibility to ensure that a nutraceutical is safe before it is marketed. The Food and Drug Administration Modernization Act of 1997 contains sections that enable health claims and nutrient content claims on food labeling to be authorized based on an authoritative statement from the Academy of Sciences or other federal authorities after notifying the FDA at least four months before the introduction of the supplement on the market [52].

The government of India established the Food Safety and Standards Act (FSSA) in 2006 to introduce a legislation system. FSSA does not separate functional foods, nutraceuticals, and dietary supplements; instead, each is indicated as food for a special dietary application. In 2015, India notified the World Trade Organization of a draft regulation for nutraceuticals and foods for special diets and medical purposes. In general, many countries, such as Australia or China, regulate nutraceuticals simply as a category of food, and the national regulations are valid for food application. Moreover, a health claim should be authorized and attributed only after a complete clinical study is proposed to the appropriate authority for approval with the aim of substantiating its safety and efficacy with respect to the claimed beneficial health effect based on an understanding of the mechanism of action and the absence of undesired side effects.

### 7.2. Impact of Placebo Effect

The impact of nutraceuticals is just like pharmaceuticals and a part of the effectiveness of nutraceuticals, which can be attributed to the placebo effect. People have used nutraceuticals as a healing illness and are often able to recover on their own. The Nobel Prize winner (Linus Pauling and Abrahm Hoffer) suggested that the provision of these nutrients might also in truth encourage the restoration mechanism; ill individuals may additionally require more nutrients to cause the mechanism [8].

## 8. Future Prospective

The increasing demand for nutraceuticals, such as food for fitness and health, is responsible for their positive and therapeutic uses for different kinds of diseases. The development and growth of new functional food or specially nutraceutical industry seem destined to occupy the landscape in the new millennium. The enzymes are used in various nutraceutical processes and play a crucial part in nutraceuticals. The next area of high consideration is the interaction between nutraceuticals and FDA. The therapeutic effectiveness of nutraceuticals remains to be determined as like drugs [11].

It is a big challenge for nutraceuticals, for the future prevention and therapy of triggering tools in the medicine area. The future possibility of nutraceuticals to prevent or support a pharmacological therapy is now recently based on pharmaceuticals, which can be a powerful tool to face pathological, chronic, and long-term diseases. The clinical study data evaluation is based on the beneficial effect of nutraceuticals, through “*in vitro* and *in vivo*” representation, which may be dispensed in an individual nutritive supplementation observed in animals [53, 54].

## 9. Conclusions

Nutraceuticals provide benefits in the prevention and treatment of various diseases. With increasing incidences of lifestyle-related health problems, they have emerged as an essential component of the diet for the common consumer. Nutraceuticals are now serving as a primary dietary supplement for health-conscious masses in India. Nutraceuticals (nutritional supplements) have fast become a staple in the healthcare market in numerous forms, including tablets, syrups, gums, and capsules. The combined and concerted action of nutrient and biologically active compounds is flagged as an indicator of a possible beneficial role for health. Nutraceutical use is growing fast and is well accepted by people for its all-natural origin. The demand for fewer synthetic pharmaceuticals is triggering this interest and stimulating also the industry to develop and put on the market new products which claim beneficial health effects. Nutraceuticals cannot replace pharmaceuticals but can be a strong high-value tool for prevention and aid in therapy of some pathological conditions. The present review provides comprehensive knowledge about all these aspects related to nutraceutical sources, formulations, scopes, challenges, quality control, stability, and safety evaluation in brief.

## Figures and Tables

**Figure 1:** Some of the important bioactive phytonutrients.

**Figure 2:** Clinical condition involving reactive oxygen species.

**Table 1:** Nutraceutical foods and their therapeutic uses.

Nutraceutical/nutrients	Therapeutic uses	References
Ketogenic/Atkins diets (high protein and fat diet with low carbohydrates)	Benefits against diabetes, cancer, epilepsy, and Alzheimer's disease	[55, 56]
Minimally refined grains, cereals, and fortified grains	Reduce diabetes, prevent gastrointestinal cancers	[57]
Phytoestrogens (soya flour and linseeds)	Enhance estrogen levels, prevent hot flushes & cancers	[57]
Edible mushrooms (Tonnage, Lentinus, Pleurites, Auricularia, Flammulina, Tremella, Hericium, & Grifola)	Immunomodulatory, lipid-lowering, and antitumor activity	[58]
Glucosamine sulfate and chondroitin sulfate	Osteoarthritis	[59]
Peptides/hydrolysates (casein, buckwheat proteins, & whey proteins)	ACE inhibitor, reduce cholesterol and hypertension, improve constipation & obesity	[60]
Dairy foods/bio yoghurts (probiotics, Lactobacillus acidophilus, & Bifidobacterium)	Promote gut health,	[61]
Fatty acids (LCPUFAs)	Important for foetal & infant development	[62]

**Table 2:** Essential micro- or macronutrients/vitamins and their therapeutic uses.

Vitamins	Therapeutic uses
Vitamin A	Maintain healthy skin, mucus membrane and vision, body growth and development, anticancer, skin disorder, and antioxidant
Vitamin D	Formation of teeth and bones (which helps the body to absorb and use calcium)
Vitamin E	Boost the immune system, antioxidant (formation of nerve tissue, blood cells, muscles, and lungs)
Vitamin K	Clotting of blood
H_2_O (soluble vitamins & acids)	
Vitamin C	Maintain good skin, gums, bones, & teeth, wound healing & reduce cold & cough, antioxidant
Vitamin B1	Essential in neurological functions and convert food into energy
Vitamin B2	Energy production, maintain healthy skin, eyes, & nerve
Vitamin B3	Convert food into energy and maintain brain function
Vitamin B6	Produce proteins and convert protein into energy
Vitamin B12	Produce the DNA of cells, form red blood cells, maintain CNS and amino acid synthesize, metabolism of fats, proteins, and carbohydrates
Folic acid	Essential for preventing birth defects, formation of RBC (“red blood cell”), produce DNA of cells, heart disease protector
Pantothenic acid	Cholesterol, fatty acids & steroid synthesis, acetylcholine intraneuronal synthesis
Vitamin-like compounds	
Biotin	Used in different biotransformation processes
L-Carnitine	Formation of certain organic acid excretion and phosphorylation, fatty acid oxidation
Choline	Lipotropic agent; these are used for treatment of fatty liver and interrupted fat metabolism
Vitamin F	Synthesis of prostaglandins, leukotrienes & different hydroxyl fatty acids, membrane development
Inositol lipotropic agents	Formation & movement of potassium & sodium, transportation of amino acid
Taurine	Conjugation of bile acid, CNS neuromodulation, retinal photoreceptor activity, antioxidant activity in WBC, platelet aggregation, cardiac contractility, sperm growth & motility, insulin growth & development activity

**Table 3:** Minerals and their therapeutic uses.

Minerals	Therapeutic uses
Macronutrients (major minerals)	
Calcium (Ca)	Development of teeth & bones, maintain bone strength, nerve, muscle, and glandular functions
Magnesium (Mg)	Nerve, muscle & bone formation, help to “prevent premenstrual syndrome (PMS)”
Phosphorous (P)	Build strong bones and teeth, formation of gene material, energy production & storage
Sodium (Na)	Nerve transmission, proper fluid balance, muscle contraction
Chloride (Cl)	Fluid balance & stomach acid
Potassium (K)	Nerve transmission & muscle contraction
Sulfur (S)	Found in protein molecules
Microelements (trace minerals)	
Chromium (Cr)	insulin helps to convert carbohydrates & fats into energy
Iron (Fe)	Energy production by carrying oxygen to tissues
Cobalt (Co)	Essential for vitamin B12, formation of B12 coenzymes
Copper (Cu)	Production of hemoglobin & collagen, healthy functioning of heart, energy production, absorption of iron from digestive tract
Iodine (I)	Thyroid functioning
Selenium (Se)	Antioxidant, essential for heart muscle functioning
Zinc (Zn)	Cell reproduction, child growth & development, wound healing, production of sperm & testosterone
Fluoride (F)	Formation of bones & teeth and prevent tooth decay

## Data Availability

The data used to support the findings of this study are available from the corresponding authors upon request.

## Abbreviations

ALA: *α*-Linolenic acid
BBB: Blood-brain barrier
CHD: Coronary heart disease
COMT: Catechol-O-methyl transferase
CoQ-10: Coenzyme Q-10
DNA: Deoxyribonucleic acid
DSHEA: Dietary Supplements Health and Education Act
FAO: Food and Agricultural Organization
FDA: Food and Drug Administration
FSSA: Food Safety and Standards Act
LA: Linoleic acid
LDL: Low-density lipoprotein
MDPI: Multidisciplinary digital publishing institute
MOA: Mechanism of action
MUFA: Monounsaturated fatty acids
NK cell: Natural killer cell
PubMed: Public/publisher Medline
PUFA: Polyunsaturated fatty acids
SciELO: Scientific electronic library online
TNF: Tumor necrosis factor
UTI: Urinary tract infection
Vita: Vitamin
WHO: World Health Organization.
